The article "Is early intervention using Mansoura-VV uterine compression sutures an effective procedure in the management of primary atonic postpartum hemorrhage? : a prospective study" was retracted in 2023. Reason: lack of ethics approval or compliance.

# Is early intervention using Mansoura-VV uterine compression sutures an effective procedure in the management of primary atonic postpartum hemorrhage? : a prospective study

**DOI:** 10.1186/s12884-017-1349-x

**Published:** 2017-05-31

**Authors:** Abd Elaziz A. El Refaeey, Hosam Abdelfattah, Alaa Mosbah, Anas M. Gamal, Emad Fayla, Waleed Refaie, Abdelhady Zaied, Rafik I. Barakat, Amal K. Seleem, Mohammed Maher

**Affiliations:** 1 Department of Obstetrics and Gynecology, Mansoura University, Mansoura, 35511 Egypt; 2 Department of Medical Biochemistry, Mansoura University, Mansoura, Egypt; 3 Department of Anesthesia, Mansoura University, Mansoura, Egypt

**Keywords:** Atonic postpartum hemorrhage, Uterine compression sutures

## Abstract

**Background:**

Postpartum hemorrhage is the leading cause of maternal death, uterine atony accounts for 75-90% of primary postpartum hemorrhage. The efficacy of the Uterine compression suture in the treatment of atonic postpartum hemorrhage is time-tested and can be said to be almost established.The aim of this study was to assess the role of the Mansoura-VV uterine compression suture as an early intervention in the management of primary atonic postpartum hemorrhage.

**Methods:**

This prospective observational study included 108 women with primary atonic PPH over a period of 44 months. Uterine atony was diagnosed when the uterus was soft and failed to respond to ordinary ecbolics. Early intervention by Mansoura-VV uterine compression sutures was carried out within 15 min of the second dose of ecobolics and before progressing to any further surgical procedure.

**Results:**

Following the Mansoura-VV uterine compression sutures, uterine bleeding was controlled in all except one patient (107/108 cases; 99.07%) who required additional bilateral uterine vessels ligation. Another case (0.93%) was subjected to re-laparotomy due to intraperitoneal hemorrhage. Packed RBC transfusion was needed in 10 cases (9.25%). Admission to ICU was needed in 9 cases (8.33%) because of associated medical conditions. One week following the procedure, 1 case (0.93%) was diagnosed with haematometra.

**Conclusion:**

Early intervention in cases of primary atonic PPH using the Mansoura-VV uterine compression sutures is an easy, rapid and effective method in controlling PPH in low resource settings.

**Trial registration:**

The study was registered at clinicaltrial.gov, Identifiers: NCT03117647 “retrospectively registererd” registered at April 7, 2017.

## Background

Worldwide, postpartum hemorrhage (PPH) is the leading cause of maternal death, with an estimated mortality rate of 140, 000 per year, or 1 maternal death every 4 min [1]. Non-fatal PPH results in further interventions, pituitary infarction with associated poor lactation, exposure to blood products, coagulopathy, iron deficiency anemia, and organ damage with associated hypotension and shock [2]. Uterine atony accounts for 75-90% of primary PPH [3]. The corner stone of effective treatment of PPH remains rapid diagnosis, realistic estimation of the amount of blood loss and prompt interventions. Treatment of PPH comprises bi-manual or mechanical compression of the uterus, uterotonic drugs and surgical methods, combined with resuscitative measures [4].

The article "Is early intervention using Mansoura-VV uterine compression sutures an effective procedure in the management of primary atonic postpartum hemorrhage? : a prospective study" was retracted in 2023. Reason: lack of ethics approval or compliance.

The majority of maternal deaths occur within 4 h of delivery [5]. Also, delay of 2–6 h between delivery and uterine compression suture (UCS) was independently associated with a four-fold increase in the odds of hysterectomy [6].

Atonic uterus is one of the preventable causes of PPH, prophylactic strategies has been adopted, the active management of the third stage of labor and intravenous or intramuscular injection of oxytocin [7]. Misoprostol has emerged as a cheap alternative drug but the results were inferior to oxytocin, with more side effects. Overall, drug treatment fails to work in less than 1% of patients [8].

The efficacy of the UCS in the treatment of atonic PPH is time-tested and can be said to be almost established [9]. Prevention of PPH is of crucial importance particularly where there is high prevalence of anemia, for even a modest PPH may lead to serious and life threatening complications. B-Lynch in his original article in 1997, stated that the cost-effectiveness of this procedure may consider its application when necessary both for prophylactic and therapeutic purposes in developing countries [10]. Although the gained world-wide popularity of the B-Lynch suture, only few reports addressed its use as a prophylactic measure in women with atonic PPH. Elective B-lynch suture has been reported successful in a parturient patient with congenital heart disease [11] as well as a pilot study on seven cases at risk of PPH during emergency CS, was successful in all cases [12].

There is limited data regarding the prophylactic or early use of the numerous UCS in the management of atonic PPH. Our novel Mansoura-VV uterine compression suture was successful in 18 out of 19 cases (94.7%) of intractable atonic PPH [13]. In this report, we expanded our experience to the application of the Mansoura-VV uterine compression suture as an early intervention procedure in women with primary atonic PPH before the patients^,^ general condition deteriorate, particularly in CS.

## Methods

This prospective observational study was carried out at the Obstetrics and Gynecology Department Mansoura University Hospital, and private settings in Mansoura, Egypt, during the period from May 2013 to December 2016. The study was approved by Institutional research board Code number: R/16.09.55.

The article "Is early intervention using Mansoura-VV uterine compression sutures an effective procedure in the management of primary atonic postpartum hemorrhage? : a prospective study" was retracted in 2023. Reason: lack of ethics approval or compliance.

Inclusion criteria included women diagnosed with primary atonic PPH, during cesarean section when the uterus failed to contract after the routine doses of uterotonics. Women and their partners were counseled and signed a consent regarding the technique as an alternative to devascularization or hysterectomy. Exclusion criteria included patients with placenta previa complete or incomplete centrails, and/or placenta accreta. Also one case of atonic PPH, when the uterus was incompressible and failed to contract on bimanual compression was excluded from the study, as in our experience these cases failed to respond to any type of UCS.

In this series, immediately after anesthesia, all women received misoprostol 400 mcg (two tablets of Misotac^R^, Adwia Co, 6th October city, Egypt) sublingual, as well as 20 IU of oxytocin (Syntocinon, Sanofi Aventais, Egypt) in 50 0-mL lactated Ringer’s solution as an intravenous infusion, after delivery of the baby and clamping of the umbilical cord. This is routine practice for all women undergoing CS in our department.

After closure of the uterine incision, uterine atony was diagnosed in 108 women when the uterus felt soft and flappy, and failed to respond to intermittent fundal massage, the second dose of the previously mentioned ecbolics was given. Then, bimanual compression of the uterus was attempted for 10 to 15 min until the tone of the uterus is regained as well as to assess the potential chances of success of the Mansoura-VV uterine compression suture.

Within 15 min of the diagnosis, the uterus was rechecked to identify any bleeding points. We performed Mansoura-VV uterine compression suture (Fig.1). **The right V** was performed as follow: (i) 100-cm Vicryl no. 1 was thrown to form two nearly equal parts (each 50 cm) on a blunt semicircular 70-mm needle, the curve of the needle was straightened. (ii) The needle transfixed the right uterine wall from anterior to posterior, about 2 cm below the hysterotomy incision and 3 cm from the (this represents the apex of the V suture) (Fig. 1a,b). (iii) after transfixation, the Vicryl was divided thus two threads from one transfixation each 50-cm threads penetrated the lower uterine segment; medial (M) and lateral (L) threads, each has anterior (aL and aM) and posterior (pL and pM) ends in relation to the uterus (Fig 1c) (iv) The free anterior and posterior ends of the lateral thread (aL and pL) were tied above the fundus with three double - throw knots about 3 cm from the right cornual border of the uterus forming the lateral limb of the V suture (Fig 1d). (v) The free anterior and posterior ends of the medial threads (aM and pM) were tied above the fundus 2–3 cm medial to the lateral limb completing the V suture (Fig 1e). The lead surgeon pulled the suture to provide moderate tension, while the assistant surgeon lift the uterus upward while perform a bimanual uterine compression to minimize trauma and to achieve or aid compression during the ligation of each vertical limb. (vi) using a similar technique, the **left V** suture was laid on the left side, and then the VV suture is completed (Fig 1f).

The article "Is early intervention using Mansoura-VV uterine compression sutures an effective procedure in the management of primary atonic postpartum hemorrhage? : a prospective study" was retracted in 2023. Reason: lack of ethics approval or compliance.

**Fig. 1:** Schematic representation of the Mansoura-VV compression sutures: A100 cm catgut no 2 was thrown to form 2 equal parts (each 50 cm) on a blunt straightened semicircular 70-mm needle. The needle transfixes the right uterine wall from anterior to posterior, about 2 cm below the hysterotomy incision (**a**, **b**). After transfixation, the cat gut was divided into 2 longitudinal medial (M) and lateral (L) threads (**c**). The free (aL and pL) ends of the lateral threads tied above the fundus about 3 cm from the right cornual border forming the lateral limb of the V suture (**d**). 5-The free ends of the medial threads (aM and pM) were tied above the fundus 2–3 cm medial to the lateral limb completing the V suture (**e**). Using a similar technique, another V suture was laid on the left side, and then the VV suture is complete (**f**)

The vagina was inspected to check for control of bleeding with Mansoura-VV sutures, the uterus cannot be stretched. Only one case (1/108) required additional bilateral uterine vessels ligation for control of bleeding, the abdomen was closed routinely. Antibiotics were given and continued postoperatively for 5 days.

## Results

Demographic parameters and baseline data included the patients’ age, number of previous deliveries, gestational age at delivery, history of prior CS, and both preoperative and 24 h postoperative hemoglobin and hematocrite values were measured as shown in Table 1. The mean maternal age was 29.2 ± 5.01 year, and the mean gestational age at termination was 37.5 ± 3.9 weeks. The median parity and number of prior CS was 3. There was no statistically significant difference (*p* > 0.05) between the mean preoperative hemoglobin levels was 11.8 ± 0.74 g/dl, and the mean postoperative hemoglobin 10.9 ± 0.53 g/dl. Similarly, there was no statistically significant difference (*p* > 0.05) between the mean preoperative hematocrite 34.9 ± 2.19 and the mean postoperative hematocrite 32.8 ± 1.58.

**Table 1:** Demographic characteristics of patients (108 cases)

	Range	Mean + SD	Median	P
Maternal age (yr)	19-42	29.2 ± 5.01	29	
Body mass index (kg/m^2^)	23-40	26.8 ± 5.01	26.7	
Gestational age at delivery (wk)	34 -41	37.5 ± 3.9	38	
Parity (no)	1- 6	2.07 ± 1.19	2	
No of prior CS	0-5	1.06 ± 1.04	1	
Hemoglobin (gm/L)				
-Preoperative	10.1-13.9	11.8 ± 0.74	11	<0.05
-Postoperative	9.1- 12.1	10.9 ± 0.53	11	
Hematocrite (%)				
-Preoperative	29-42	34.9 ± 2.19	35	<0.05
-Postoperative	28-39	32.8 ± 1.58	33	

*P* value >0.05 is significant

The indications of CS were multiple pregnancy (24 cases), fetal macrosomia (17 cases), preclampsia/Eclampsia (12 cases), arrest of cervical dilatation (17 cases), abruptio-placenta (10 cases), polyhydramnios (9 cases), anterior or posterior placenta previa (9 cases), rheumatic heart diseases (8 cases), and acute fetal distress (2 cases) presented in Table 2.

The article "Is early intervention using Mansoura-VV uterine compression sutures an effective procedure in the management of primary atonic postpartum hemorrhage? : a prospective study" was retracted in 2023. Reason: lack of ethics approval or compliance.

**Table 2:** Indications of cesarean sections (*n* = 108 women)

	No	Percent
-Multiple pregnancy	24	22.2%
-Fetal macrosomia	17	15.7%
-Arrest of cervical dilatation	17	15.7%
-Preclampsia/Eclampsia	12	11.1%
-Abruptio placenta	10	9.3%
-Placenta previa (anterior or posterior)	9	8.3%
-Polyhydramnios	9	8.3%
-Rheumatic heart diseases	8	7.4%
-Acute fetal distress	2	1.9%
-Total no of cases	108	100%

Hemostasis and adequate uterine compression was achieved after applying Mansoura-VV uterine compression suture in all cases except one (99.07%). In one case of atonic PPH with placenta previa bleeding was controlled after bilateral ligation of the uterine vessels and additional vertical compression sutures in the lower uterine segment was performed. Moreover, none of the 108 patients required hysterectomy. Re-laparotomy was done for one patient, there was intraperitoneal hemorrhage from the uterine incision and venous plexus in the utero-vesical pouch, it was controlled by hemostatic sutures, and bilateral ligation of uterine arteries. Transfusion of red blood cells (RBC), admission to ICU, postoperative fever, hematometra were shown in Table 3.

**Table 3:** Intra and post-operative complications and follow up

	No	Percent
Intra-operative complications		
-Additional uterine vessels ligation and vertical sutures in the lower uterine segment	1	0.93%
-Hysterectomy	0	0
Immediate complications		
-Blood transfusion	10	9.26%
-Admission to ICU	9	8.33%
Minor complications		
Post-operative fever	7	6.48%
-Hematometra	1	0.93%
-Short term follow-up period		
Followed-up to 1 week	108	100%
Followed-up to 4 weeks	94	87%
Followed-up to 6 weeks	80	74.07%

Transfusion of RBCs were given to 10 women out of 108 (9.25%), admission to ICU was done for 9 cases (8.33%), During follow up minor complications as postoperative fever was identified in 7 cases (6.48%), one case was diagnosed with hematometra diagnosed on the 7th postoperative day.

The article "Is early intervention using Mansoura-VV uterine compression sutures an effective procedure in the management of primary atonic postpartum hemorrhage? : a prospective study" was retracted in 2023. Reason: lack of ethics approval or compliance.

During the follow up period, 20 women (18.51%) conceived, spontaneous abortion occurred in 2 cases (10%). Among the 16 women who gave birth, 3 had vaginal birth after cesarean section, 13 women were delivered by repeat CS. At the time of writing this work, there are ongoing 2 pregnancies.

Descriptive statistics were used to examine maternal age, BMI, parity, number of previous CS and gestational age. The statistical analysis was performed using SPSS package (version 18; SPSS Inc., Chicago, Il). Discrete data were analyzed with analysis of variance test (ANOVA). *P* < 0.05 was considered significant throughout.

## Discussion

In 2010, we used our innovative technique; the Mansoura-VV uterine compression suture to treat intractable PPH during CS who did not respond to mechanical/ecobolic treatments at our institution, it was successful in 94.7% [14]. We experienced a learning curve and tried to use the same technique at an earlier stage in the course of management of atonic PPH to prevent the maternal near misses and before deterioration of the patient’s general condition.

The aim of the present study was to assess the role of Mansoura-VV uterine compression suture as an early intervention technique in cases of atonic PPH encountered during CS, and before deterioration of the patient’s general condition. The Mansoura-VV uterine compression suture was performed in 108 cases delivered by CS; when the uterus felt soft, flappy, and failed to respond to the second dose of uterotonics. Application of Mansoura VV uterine compression suture within 15 min was successful in controlling the uterine bleeding in all except one case (99.07%).

To the best of our knowledge, this is the largest case series using an early intervention in cases of atonic PPH. Although, the efficacy of the uterine compression sutures (UCS) is difficult to evaluate, our results compare favorably with the results reported by Vachhani and Virkud 2006, who conducted a pilot study on 7 cases at risk of PPH subjected to the B-Lynch and reported a successful outcome in all cases [12]. Our results were higher than that reported by Kayem et al., [6] who performed a meta-analysis on the UK Obstetric Surveillance System and concluded that the use of UCS within 1 h after delivery yielded a higher success rate of 84% [6]. This difference in the results may be explained by differences in UCS techniques, as well as differences in the timing of the UCS as some institutes may employ the uterine compression suture at the last moment of very severe PPH, while other institutes may employ the sutures in less severe situations [9].

The mechanism for control of atonic uterine bleeding using Mansoura-VV uterine sutures, probably is due to the marked reduction of the uterine blood flow through the lateral arms of the sutures, as well as compression of the placental site. The added medial arms of the suture may add an extra pillar to compress the central portion of the uterus more effectively. The Mansoura-VV uterine sutures has some advantages, that it avoids the necessity of re-opening the uterine incision as in the original B-Lynch, more effective compression of the uterus, fewer needle bites, and better drainage of the uterus as we explained previously [13].

The article "Is early intervention using Mansoura-VV uterine compression sutures an effective procedure in the management of primary atonic postpartum hemorrhage? : a prospective study" was retracted in 2023. Reason: lack of ethics approval or compliance.

The main target of the Mansoura-VV suture compression sutures was to control uterine bleeding from atony, yet, the suture worked successfully in 8 out of 9 cases (88.88%) with placenta previa. This high success rate may be attributed mainly to the proper surgical technique and partly to the exclusion of cases of placenta accreta. In only one case (1 out of 9) of anterior placenta previa, uterine bleeding was controlled by additional bilateral uterine vessels ligation and multiple vertical compression sutures through the full thickness of the anterior and posterior uterine walls in the lower uterine segment. This denotes that even in cases of placenta previa, early intervention using Mansoura-VV uterine compression suture could be used as a first aid measure to reduce the degree of hemorrhage and to avoid the adverse consequences of severe hemorrhage. None of the 108 patients required hysterectomy,

Admission to ICU needed in 9 cases (9.9%), due to the presence of associated conditions such as preeclampsia/eclampsia, rheumatic heart disease, abruptio placenta. During follow up, minor complications were observed such as postoperative fever in 7 cases (6.48%), wound sepsis in 4 cases. Obviously these were not due to the procedure itself. On the 7th postoperative day, one case was diagnosed with hematometra and was subjected to evacuation under general anesthesia. It remains to be established whether opening of the cervix at the time of elective CS, prevents the development of hematometra or not in cases where UCS were done.

There were no observed cases of pyometra after the Mansoura VV uterine sutures, contrary to what was reported in some types of other compression sutures [14], this may be due the fact that the uterine cavity was not re-opened during the procedure that may reduce the incidence of endometritis or sepsis. Normal menstrual patterns were resumed in 94 women out of 108 after having VV uterine compression suture, this were in accordance with our previous report [14] and with others [15].

These good results may encourage obstetricians particularly in developing countries with low resource settings to consider early intervention using Mansoura-VV uterine compression suture as an easy and low cost technique in poor resource countries where limited blood banking, lack of rapid transportation, the non availability of a 24 h trained obstetrician, and possibly infrequent availability of relatively expensive and more effective uterotonics as carbetocin or carbnaprost F_2α_.

The article "Is early intervention using Mansoura-VV uterine compression sutures an effective procedure in the management of primary atonic postpartum hemorrhage? : a prospective study" was retracted in 2023. Reason: lack of ethics approval or compliance.

## Conclusion

Early intervention in cases of atonic PPH using the Mansoura-VV suture is a simple, highly effective, and is a less time consuming procedure. It seems safe, inexpensive, and has low incidence of minor complications.

## Abbreviations

CS: Cesarean section
ICU: Intensive care unit
PPH: Postpartum hemorrhage
UCS: Uterine compression suture
UK: United Kingdom
